The article "Study on the Changes and Significance of Immune State and Cycokines in Children with Adenovirus Pneumonia" was retracted in 2023. Reasons: signs of a paper mill; suspected computer-generated content; unreliable results or conclusions; concerns about the data.

# Study on the Changes and Significance of Immune State and Cycokines in Children with Adenovirus Pneumonia

**DOI:** 10.1155/2022/2419454

**Published:** 2022-09-02

**Authors:** Yue Hou, Jing Liu, Yanan Li, Fang Chen

**Affiliations:** Department of Traditional Chinese Medicine, Beijing Children's Hospital, Capital Medical University, National Center for Children's Health, Beijing 100045, China

## Abstract

**Objective:**

To observe the difference between peripheral blood T lymphocytes subsets and cycokines in children with severe adenovirus pneumonia and nonsevere adenovirus pneumonia, and to investigate their clinical value in the prognosis of severe pneumonia.

**Methods:**

215 children with adenovirus pneumonia and 30 healthy volunteers (which was set as the control group) in our hospital from January 2017 to May 2019 were enrolled in the study. There were 47 children with severe pneumonia in the severe group and 168 nonsevere pneumonia children in the nonsevere group. The flow cytometry and ELISA methods were used to detect the serum levels of CD_3_^+^, CD_4_^+^, CD_8_^+^ T cells and interleukin-2 (IL-2), IL-4, IL-6, IL-10, tumor necrosis factor-*α* (TNF-*α*), interferon-*γ* (IFN-*γ*).

**Results:**

(1) The levels of CD_3_ (%) T cells, CD_4_ (%) T cells, and CD_4_/CD_8_ ratio values of children with adenovirus pneumonia were lower than these of normal children (*P* < 0.05). And the levels of CD_3_ (%) T cells, CD_4_ (%) T cells, and CD_4_/CD_8_ ratio values of children in the severe group were lower than these of children in the nonsevere group (*P* < 0.05). (2) The levels of IL-2, IL-6, IL-10, TNF-*α,* and IFN-*γ* values of children with adenovirus pneumonia were lower than these of normal children (*P* < 0.05). And the levels of IL-2, IL-6, IL-10, TNF-*α,* and IFN-*γ* of children in the severe group were higher than these of children in the nonsevere group (*P* < 0.05). (3) Among the 47 children with severe adenoviral pneumonia, 39 received systematic treatment in our hospital. According to the treatment effect, 39 children were divided into the effective group (*n* = 25) and the ineffective group (*n* = 14). (4) The CD3 (%), CD4 (%), and CD4/CD8 ratios of the children in the effective group were higher than those in the ineffective group (*P* < 0.05). (5) The levels of IL-2, IL-6, IL-10, TNF-*α,* and IFN-*γ* in the effective group were lower than those in the ineffective group (*P* < 0.05).

**Conclusion:**

The immunophenotype of peripheral blood T lymphocytes and cycokines could be helpful to judge the severity of adenovirus pneumonia, which could be used as the objective indexes to evaluate the prognosis of children with severe adenovirus pneumonia.

The article "Study on the Changes and Significance of Immune State and Cycokines in Children with Adenovirus Pneumonia" was retracted in 2023. Reasons: signs of a paper mill; suspected computer-generated content; unreliable results or conclusions; concerns about the data.

## 1. Introduction

Adenovirus is one of the most important pathogens causing severe pneumonia in children, and it is easy to cause multisystem complications. It is one of the main causes of death of an infant under 2 years old [1], which greatly increases the social medical burden. The onset of adenovirus pneumonia is acute, usually manifesting obvious symptoms of pneumonia 4-5 days after fever, and the course of the disease can be prolonged for several months, which can eventually lead to bronchiectasis, chronic obstructive pulmonary disease, and even death. However, due to the lack of typical clinical indications in the early stage, severe pneumonia can only be diagnosed when typical severe hypoxia, sepsis, and multiple organ dysfunctions occur, resulting in a high mortality rate in children [2]. Therefore, it is very important to find sensitive biomarkers to reflect the degree of disease progression as soon as possible and objectively for clinical individualized treatment and improving the prognosis of children with adenovirus pneumonia. As early as the 1970s, some scholars proposed that the lung tissue damage caused by adenovirus may be involved in immunological mechanisms [3]. In addition, adenovirus infection also involves a variety of inflammatory cells and inflammatory mediators. Chemokines and cytokines are the most important messengers of the immune system and play an important role in maintaining the balance of immune responses [4]. If an immune imbalance occurs in the body, it may cause uncontrolled pulmonary inflammatory responses, resulting in multiple organ dysfunctions. This study intends to observe the immune typing of peripheral blood lymphocytes and differential changes in the levels of interleukin-2 (IL-2), IL-4, IL-6, IL-10, tumor necrosis factor-*α* (TNF-*α*), and interferon-*γ* (IFN-*γ*) in children with severe adenovirus infection to explore the infection mechanism of adenovirus from cytokine levels and whether it can help early diagnosis and prognosis prediction of severe adenovirus pneumonia. The research is reported as follows.

## 2. Materials and Methods

### 2.1. General Information

This study selected 215 children with pneumonia who were hospitalized in the Pediatrics Department of our hospital from January 2017 to May 2019. They were admitted to the hospital due to fever, cough, shortness of breath, chest tightness, dyspnea and other reasons. Among them, 126 were male and 89 were female, ranging in age from 2 months to 8 years, with an average age of (39.27 ± 10.62) months. Inclusion criteria: (1) Admission to the hospital within 3 days of acute onset; (2) Age ≤ 8 years old; (3) Meet the relevant diagnostic criteria of adenovirus pneumonia, the child developed acute fever, accompanied by respiratory, nervous, digestive and circulatory symptoms, their adenovirus was detected by respiratory immunofluorescence technique, the antigen was positive and/or the adenovirus PCR was positive [5]; (4) Complete clinical data and treatment process. Exclusion criteria: (1) Associated with other respiratory diseases such as bronchial asthma, pulmonary *tuberculosis*, malignant tumor; (2) Associated with definitely diagnosed immune system diseases; (3) Took glucocorticoids or immunosuppressants for nearly 3 months. According to the diagnostic criteria for severe pneumonia in the Guidelines for the Management of Community-Acquired Pneumonia in Children (2013 Revised Edition) issued by the Respiratory Group of the Pediatric Branch of the Chinese Medical Association in 2013 [6], they are divided into the severe group (*n* = 47) and the nonsevere group (*n* = 168) according to the severity of their illness. Infants with an axillary temperature greater than 38.5 C, poisoning symptoms, repeated high fever, more than 70 breaths per minute, older infants with a temperature greater than 38.5 C, and more than 50 breaths per minute, or complicated with any one of multiple organ function impairment, heart failure, respiratory failure, and shock, all of which can be considered as severe pneumonia.. In addition, 30 healthy children (whose age and gender ratio were matched with those of children with severe pneumonia) from the Pediatrics Department of our hospital during the same period were selected as the control group. This study complies with medical ethics requirements, and informed consent was signed by the families of the patients. There was no significant difference in general clinical data such as age, gender composition, and premature infants among the three groups (*P* > 0.05), as shown in Table 1.

The article "Study on the Changes and Significance of Immune State and Cycokines in Children with Adenovirus Pneumonia" was retracted in 2023. Reasons: signs of a paper mill; suspected computer-generated content; unreliable results or conclusions; concerns about the data.

### 2.2. Treatment

All the enrolled children were treated with antiviral therapy after admission and kept the airway open; children with bacterial infections need to be treated with antibiotics, and comprehensive supportive treatment was given according to the symptoms of the children, such as oxygen inhalation, sedation, and fever reduction, relieving spasm and asthma, relieving panic and protecting the organs, actively responding to the accompanying complications, and giving mechanically assisted ventilation to critically ill children.

### 2.3. Detection Indicators

Collection of blood samples: Blood samples of all the enrolled children were taken the next day after admission, 2 mL of fasting venous blood from children in the morning was aseptically drawn by pediatric professional nurses, and centrifuged at 3000 r/min for 10 min. The serum was taken and stored in a −80°C refrigerator for testing.

Detection of T cell subsets determined by flow cytometry. We added 100 *μ*L of anticoagulant and 20 *μ*L of RD1-CD_4_, ECD-CD_8_, and PE-CD_3_ fluorescently labeled monoclonal antibodies and isotype control antibodies. We added 500 *μ*L of hemolysin and acted for 20 min at room temperature in the dark. After lysing the red blood cells, we added a fixative for fixation. The proportion of positively expressed cells was calculated by MultiSET software, the negative control was used as the background parameter, the fluorescence compensation was adjusted, and the positive parameter value was set to obtain the proportion of each lymphocyte subsets CD_3_, CD_4_, and CD_8_ and calculate the CD_4_/CD_8_ ratios. The MultiTEST kit was provided by BD Company in the United States.

Detection of inflammatory factors-related indicators (IL-2, IL-4, IL-6, IL-10, TNF-*α*, and IFN-*γ*) were detected by the ELISA antibody double sandwich method. Took out the kit and specimen from the refrigerator 20 minutes in advance and equilibrate to room temperature. We shook all reagents well before use and diluted the standards to different concentrations. We added the samples and standards of different concentrations (100 *μ*L per well) to the corresponding wells and mark them. We strictly followed the operating instructions for testing and duplicated wells for samples (including standards) and blank wells. ELISA detection kits were purchased from Shanghai Jimian Industrial Co., Ltd.

### 2.4. Statistical Processing

The data were input into SPSS17.0 statistical software for processing and analysis; the measurement data were expressed as ($\bar{\chi }$ ± *s*); the data between two groups were compared by *t*-test; the data comparison between multiple groups was analyzed by one-way ANOVA; and the enumeration data were expressed as (%), and *χ*^2^ test was used. *P* < 0.05 was considered to be statistically significant.

## 3. Results

### 3.1. Comparison of Immune Typing of Peripheral Blood Lymphocytes in Children Tested

Comparing the peripheral blood CD_3_ (%), CD_4_ (%), and CD_4_/CD_8_ ratios of the three groups of children, the variance analysis showed that the difference was statistically significant (*P* < 0.05). Compared with the control group, the CD_3_ (%), CD_4_ (%), and CD_4_/CD_8_ ratios of the children with adenovirus pneumonia were lower, Moreover, the peripheral blood CD_3_ (%), CD_4_ (%), CD_8_ (%), and CD_4_/CD_8_ ratios of the children in the severe group were lower than those in the nonsevere group, as shown in Table 2.

### 3.2. Comparison of Peripheral Blood Cytokine Levels in Children

The serum levels of IL-2, IL-6, IL-10, TNF-*α,* and IFN-*γ* were compared among the three groups, and the variance analysis showed that the differences were statistically significant (*P* < 0.05). Compared with the control group, the levels of IL-2, IL-6, IL-10, TNF-*α,* and IFN-*γ* in the children with adenovirus pneumonia were increased, and the levels of IL-2, IL-6, IL-10, TNF-*α*, and IFN-*γ* of the children in the severe group were higher than those in the nonsevere group. In addition, the levels of IL-4 in the peripheral blood of the three groups of children were basically the same, and the difference was not statistically significant (*P* > 0.05), as shown in Table 3.

The article "Study on the Changes and Significance of Immune State and Cycokines in Children with Adenovirus Pneumonia" was retracted in 2023. Reasons: signs of a paper mill; suspected computer-generated content; unreliable results or conclusions; concerns about the data.

### 3.3. Treatment Results of Children with Severe Adenovirus Pneumonia

All children with severe adenovirus pneumonia were hospitalized for 7–45 days, with an average hospitalization of (18.43 ± 9.04) days. Among 47 children with severe adenoviral pneumonia, 39 children were treated with an auxiliary ventilator, and 8 children were not cured and discharged (their parents gave up treatment). The prognosis of 39 treated children after discharge is as follows There were 17 patients (43.59%) and 8 patients (20.51%) who were clinically cured and clinically improved, respectively, which were regarded as the effective treatment group, 14 cases (35.90%) were unhealed and died, regarded as the ineffective treatment group.

### 3.4. Differences in Immune Typing of Peripheral Blood Lymphocytes of Severe Adenovirus Pneumonia Children with Different Treatment Results

The CD_3_ (%), CD_4_ (%), and CD_4_/CD_8_ ratios of children with severe adenovirus pneumonia in the effective group and the ineffective group were compared. The CD_3_ (%), CD_4_ (%), and CD_4_/CD_8_ ratios of the children in the effective group were higher than those in the ineffective group, the difference was statistically significant (*P* < 0.05). There was no significant difference in peripheral blood CD_8_ (%) between the two groups (*P* > 0.05). See Table 4.

### 3.5. Comparison of Peripheral Blood Cytokine Levels of Severe Adenovirus Pneumonia Children with Different Treatment Results

The levels of IL-2, IL-6, IL-10, TNF-*α*, and IFN-*γ* were compared between the effective group and the ineffective group. The levels of IL-2, IL-6, IL-10, TNF-*α,* and IFN-*γ* in the effective group were lower than those in the ineffective group, the difference was statistically significant (*P* < 0.05). There was no significant difference in peripheral blood IL-4 levels between the two groups (*P* > 0.05). See Table 5.

## 4. Discussion

Adenovirus is a double-stranded DNA virus first isolated from tonsil tissue. It is one of the most common pathogens that cause respiratory tract infections in children. One-third of children with adenovirus pneumonia may develop into severe pneumonia; it is easy to combine with multisystem complications and has a high mortality rate [7]. In this study, 215 children with adenoviral pneumonia hospitalized in the respiratory department and PICU of our hospital were randomly selected, of which 47 were severe children, and the incidence of severe pneumonia was 21.86%. Moreover, most of the children were aged less than 1 year, which may be related to the lack of adenovirus-specific antibodies and low immunity in children of this age. Because most children only show clinical symptoms such as fever and cough in the early stage of adenovirus infection, a small number of children will have shortness of breath, wheezing, cyanosis, etc., and pulmonary signs often appear later, and wet rales and pulmonary consolidation signs may appear after 3 days. Therefore, most parents of children may not choose to seek medical treatment for the first time. Therefore, we chose children who sought medical treatment within 3 days of onset as the objects. The main pathological changes of adenovirus pneumonia are extensive necrosis of bronchial epithelial tissue and alveolar interstitial inflammation. In severe cases, it can lead to bronchial lumen occlusion and even lead to other system dysfunctions [8]. However, the virulence of adenovirus and its metabolites is very small. Especially in the early stage of infection, adenovirus has little effect on the survival of cells [8]. Only when the inclusion body develops to a late stage will it have a certain killing effect on the host cell. In addition, adenoviruses only parasitize in bronchial mucosal epithelial cells and lung epithelial cells [9], so relying solely on the killing effect of adenoviruses on parasitic host cells cannot explain the multiple organ damage caused by adenovirus pneumonia, especially severe pneumonia. Immunological mechanisms and cytokines may play a key role in this. Based on the author's years of clinical experience and numerous research conclusions, the damage caused by the inflammatory response caused by adenovirus pneumonia may be greater than the damage caused by the virus replication itself, which may be one of the main factors affecting the clinical severity of adenovirus pneumonia [10].

The article "Study on the Changes and Significance of Immune State and Cycokines in Children with Adenovirus Pneumonia" was retracted in 2023. Reasons: signs of a paper mill; suspected computer-generated content; unreliable results or conclusions; concerns about the data.

In this study, we first compared the differences in peripheral blood lymphocyte typing and cytokine levels between children with severe adenovirus pneumonia, children with nonsevere adenovirus pneumonia, and normal children, and planned to analyze the immunology and inflammatory response to investigate the pathogenesis of severe adenovirus pneumonia. The results of the study showed that compared with the normal control group and the nonsevere group, the peripheral blood CD_3_ (%), CD_4_ (%), CD_8_ (%), and CD_4_/CD_8_ ratios of the severe group were decreased, while the inflammatory factors of IL-2, IL-6, IL-10, TNF-*α*, and IFN-*γ* increased. It is suggested that during the acute attack of adenovirus pneumonia, the functions of CD_4_^+^T cells to promote cellular immunity and humoral immunity were significantly inhibited, and the functions of CD_8_^+^T cells to inhibit the proliferation and differentiation of immune cells were also affected. However, unlike the children with severe adenovirus pneumonia, the CD_8_^+^ T cell activity in the nonsevere adenovirus children was not statistically different from that in the normal children, and the decrease in CD_3_ (%), CD_4_ (%), and CD_4_/CD_8_ ratios did not obviously, the degree of inhibition and cytotoxicity of T cells in children with nonsevere adenovirus pneumonia was less than that in children with severe adenovirus pneumonia. Mature T cells in peripheral blood are mainly CD_3_^+^ T cells, CD_4_^+^ T cells can be divided into helper T cell 1 (Th1) subsets and Th2 subsets, while Th1/Th2 imbalance is related to viral infection. The function of CD8+ T cells is to directly kill the target antigen, mainly belonging to cytotoxic T lymphocytes, and the normal CD_4_/CD_8_ ratio maintains a dynamic balance within a certain range, but under the condition of virus infection, the CD_4_/CD_8_ imbalance, leading to immune dysfunction and reduced immune defense [11]. The CD_3_ (%), CD_4_ (%), CD_8_ (%), and CD_4_/CD_8_ ratios of adenovirus-infected children were all decreased, indicating that the body's immune function was significantly inhibited and the immune system was unbalanced, resulting in adenovirus evasion of T lymphocyte-mediated immune attack. In addition, this study also found that the proportion of T lymphocyte subsets in children with severe adenovirus pneumonia was also closely related to prognosis. The immune function of the children in the severe group declined more seriously, resulting in continued uncontrolled infection.

In addition, cytokines secreted by T lymphocytes also play an important role in immune regulation. At present, the relatively mature T cells secreting cytokines are the Th1 subset and Th2 subset [12]. Th1 cells mainly secrete IL-2 and IFN-*γ* to mediate cellular immune responses, while Th2 cells mainly secrete IL-4, IL-6, IL-10, and other factors to mediate humoral immune responses [13]. IL-2 is the most active T cell growth factor at present, IFN-*γ* is a bridge connecting innate immunity and adaptive immunity and can also enhance the antiviral effect of type I interferon, which can promote the immune function of the body after virus infection recovery. In this study, the levels of inflammatory factors such as IL-2 and IFN-*γ* in the severe group were higher than those in the control group and nonsevere group, which may be related to the feedback regulation of inflammatory factors. IL-6 and IL-10 are a class of cellular inflammatory factors secreted by Th2 cells, macrophages, vascular endothelial cells, etc., which can inhibit the activation of Th1 cells and feedback regulate the release of various cytokines including IL-2 and IFN-*γ* [14]. IL-4 belongs to a class of typical chemokines that can mediate T cell activation and has certain antiviral effects [15]. However, in this study, the levels of IL-4 in peripheral blood of the three groups are basically the same, and the test results are not statistically significant, which may be due to the small sample size. In addition, TNF-*α* is secreted by activated macrophages, NK cells, and T cells and is involved in the initiation of inflammatory responses and the regulation of immune responses. The increased TNF-*α* level leads to the infiltration of local inflammatory cells and the release of inflammatory mediators, which is closely related to the severity of the inflammatory response, and high levels of cytokines, such as IL-2 and IFN-*γ*, can promote the secretion of TNF-*α* by mononuclear macrophages [16, 17].

The article "Study on the Changes and Significance of Immune State and Cycokines in Children with Adenovirus Pneumonia" was retracted in 2023. Reasons: signs of a paper mill; suspected computer-generated content; unreliable results or conclusions; concerns about the data.

In conclusion, the peripheral blood CD_3_ (%), CD_4_ (%), CD_8_ (%), and CD_4_/CD_8_ ratios of children with severe adenovirus pneumonia were decreased, while the levels of IL-2, IL-6, IL-10, TNF- *α*, IFN-*γ,* and other cytokines all increased, indicating that the immune function of the body was suppressed. Adenovirus can evade the attack of T lymphocytes by stimulating the secretion of various cytokines, thereby strengthening the inflammatory response and causing damage to lung tissue. In addition to confirming that T cell subsets and cytokines such as IL-2, IL-6, IL-10, TNF-*α*, and IFN-*γ* are related to the severity of adenovirus pneumonia, this study is also expected to be a potential indicator for predicting the prognosis of children with severe adenovirus pneumonia.

## Figures and Tables

**Table 1:** Analysis of general data of the selected children average age.

Group	Number of children (cases)	Average age(*χ* ± *s*, month)	Gender (cases)		Preterm infants [cases (%)]	Age ≤ 12 months [cases (%)]
			Male	Female		
Control group	30	37.73 ± 9.86	16	14	2 (6.67)	7 (23.33)
Severe group	47	38.29 ± 9.49	32	15	7 (14.89)	18 (38.30)
Nonsevere group	168	39.81 ± 9.05	94	74	17 (10.12)	48 (28.57)
*F/χ* ^*2*^	—	0.592	2.519		1.444	2.344	
*P* value	—	0.554	0.284		0.486	0.310	

The article "Study on the Changes and Significance of Immune State and Cycokines in Children with Adenovirus Pneumonia" was retracted in 2023. Reasons: signs of a paper mill; suspected computer-generated content; unreliable results or conclusions; concerns about the data.

**Table 2:** Comparison of immune typing of peripheral blood T lymphocytes in children ($\bar{\chi }$ ± *s*).

Group	Number of children (cases)	CD_3_ (%)	CD_4_ (%)	CD_8_ (%)	CD_4_/CD_8_
Control group	30	67.27 ± 4.91	35.72 ± 3.79	24.45 ± 3.17	1.45 ± 0.18
Severe group	47	54.33 ± 5.26^a^	20.03 ± 5.14^a^	21.56 ± 2.91^a^	0.96 ± 0.22^a^
Nonsevere group	168	63.82 ± 6.37^ab^	31.19 ± 3.96^ab^	23.82 ± 3.40^b^	1.36 ± 0.21^ab^
*F*	—	8.859	9.512	5.228	7.041
*P* value	—	0.000	0.000	0.002	0.000

Note: Compared with the control group, ^a^*P* < 0.05; compared with the severe group, ^b^*P* < 0.05.

**Table 3:** Comparison of immune typing of peripheral blood T lymphocytes in children (pg/mL, $\bar{\chi }$ ± *s*).

Group	Number of children (cases)	IL-2	IL-4	IL-6	IL-10	TNF-*α*	IFN-*γ*
Control group	30	4.18 ± 2.33	2.54 ± 0.74	8.29 ± 2.67	8.41 ± 1.19	1.35 ± 0.67	2.84 ± 1.13
Severe group	47	94.25 ± 19.64^a^	2.62 ± 0.68	67.61 ± 10.23^a^	25.78 ± 6.34^a^	7.72 ± 2.50^a^	28.96 ± 9.49^a^
Nonsevere group	168	23.71 ± 6.95^ab^	2.55 ± 0.65	19.48 ± 5.11^b^	15.20 ± 4.72^ab^	2.41 ± 1.08^b^	11.27 ± 4.25^ab^
*F*		1001.219	0.221	1257.006	135.728	284.715	260.205
*P* value		0.000	0.802	0.000	0.000	0.000	0.000

Note: Compared with the control group, ^a^*P* < 0.05; compared with the severe group, ^b^*P* < 0.05.

**Table 4:** Comparison of immune typing of peripheral blood T lymphocytes in severe adenovirus pneumonia children with different treatment results ($\bar{\chi }$ ± *s*).

Group	Number of children (cases)	CD_3_ (%)	CD_4_ (%)	CD_8_ (%)	CD_4_/CD_8_
Effective group	25	59.24 ± 2.35	22.56 ± 2.49	21.76 ± 1.73	1.03 ± 0.12
Ineffective group	14	53.16 ± 2.71	19.02 ± 1.28	21.28 ± 2.20	0.92 ± 0.15
*t*	—	7.337	4.946	0.754	2.509
*P* value	—	0.000	0.001	0.456	0.017

**Table 5:** Comparison of peripheral blood cytokine levels of severe adenovirus pneumonia children with different treatment results (pg/mL, $\bar{\chi }$ ± *s*).

Group	Number of children (cases)	IL-2	IL-4	IL-6	IL-10	TNF-*α*	IFN-*γ*
Effective group	25	80.78 ± 9.69	2.68 ± 0.61	61.45 ± 12.38	22.17 ± 6.17	6.46 ± 1.53	19.58 ± 7.67
Ineffective group	14	108.92 ± 17.16	2.51 ± 0.48	73.22 ± 9.25	30.67 ± 4.33	10.02 ± 1.93	29.38 ± 7.96
*t*	—	6.575	0.897	3.099	4.553	6.343	3.777
*P* value	—	0.000	0.376	0.004	0.000	0.000	0.001

## Data Availability

The data used and/or analyzed during the current study are available from the corresponding author.
